The article "Construction and Drug Evaluation Based on Convolutional Neural Network System Optimized by Grey Correlation Analysis" was retracted in 2023. Reasons: unreliable results or conclusions; concerns about the data; concerns about the peer review; concerns about the citations.

# Construction and Drug Evaluation Based on Convolutional Neural Network System Optimized by Grey Correlation Analysis

**DOI:** 10.1155/2021/2794588

**Published:** 2021-09-15

**Authors:** Hui Teng

**Affiliations:** Basic Medical Science College, Qiqihar Medical University, Qiqihar, Heilongjiang 161006, China

## Abstract

Incidence rate of mental illness is increasing year by year with the development of city. The amount of modern medical data is huge and complex. In many cases, it is difficult to realize the rational allocation of resources, which puts forward an urgent demand for the artificial intelligence of modern medicine and brings great pressure to the development of the medical industry. The purpose of this study is to develop and construct a grey correlation analysis and related drug evaluation system of mental diseases based on deep convolution neural network. The establishment of the system can effectively improve the automation and intelligence of modern psychiatric treatment process. In this article, the grey correlation analysis of patient data is carried out, and then, the optimized deep convolution neural network is constructed. Combined with the medical knowledge base, the analysis of disease results is realized, and on this basis, the efficacy of related drugs in the treatment of mental diseases is evaluated. The results show that the advantage of the deep convolution neural network system is to effectively improve the induction rate. What's more, compared with other algorithms, this algorithm has higher accuracy and efficiency. It improves the comprehensiveness and informatization of disease screening methods, improves the accuracy of screening, reduces the consumption of doctors' human resources, and provides a theoretical basis for the digitization of the medical industry in the future.

## 1. Introduction

In recent years, with the development of science and technology, many breakthroughs have been made in the field of deep learning. Convolutional neural network (CNN) reported many research results that are very eye-catching [1–3]. The advantage of deep convolution neural network is not only that it can imitate the human visual system and extract image features layer by layer, which can improve the recognition rate, but also the stability and good translation invariance of these features, which can improve the accuracy of analysis and processing [4, 5]. Based on the above advantages, deep convolution neural network is widely used in many industries, including but not limited to face, image, and speech recognition [6–8].

Grey relational analysis (GRA) is a common analysis method, which is mostly used to count the influence of multiple factors on the results [9, 10]. In many cases, there are many factors affecting the process of the results, and we need to analyze which index is more relevant or the correlation ranking of these factors, and we can get the response results through the grey correlation analysis.

The article "Construction and Drug Evaluation Based on Convolutional Neural Network System Optimized by Grey Correlation Analysis" was retracted in 2023. Reasons: unreliable results or conclusions; concerns about the data; concerns about the peer review; concerns about the citations.

In recent years, with the development of society, people's demand for spiritual life is increasing, the incidence of mental illness is also increasing year by year, and the incidence is mostly concentrated in big cities [11–13]. Modern medicine has a huge amount of complex data; in many cases, it is difficult to achieve a reasonable allocation of resources, which puts forward an urgent demand for the artificial intelligence of modern medicine and also brings great pressure to the development of the medical industry [14–16]. Compared with other kinds of diseases, the medical data of mental diseases may have more complex data records, which consumes a lot of medical human resources. However, the scope of computer identification data is limited and can only be applied to structured data. Therefore, we need to process the massive data of mental diseases to construct an evaluation system that is widely used in the analysis of mental illness.

In recent years, deep learning is a very important aspect in the field of machine learning, especially in the medical and other industries [17, 18]. Machine learning relies on the process of computer recognition data, which is limited to a certain extent, and requires manpower and material resources to develop specific evaluation indicators for each mental disease [19, 20]. These indicators are special and constantly change with the types of diseases, which is not conducive to the unified processing of intelligent data [21–23]. Deep learning can integrate data and represent specific indicators of data by combining higher level features that claim to be abstract [24, 25]. Because of its good feature extraction ability and system construction method, it can be applied to many different areas of mental illness [26–28].

There is a huge space for in-depth learning and development in the medical industry, especially in the assessment of mental illness. Therefore, the purpose of this study is to develop and construct a grey relational analysis of mental illness and evaluation system of related drugs based on deep convolution neural network. The establishment of this system can effectively improve the automation and intelligence of modern psychiatric treatment process. In this article, the grey correlation analysis of the patient data was carried out and then construction of the optimized depth convolution neural network was done, combined with the medical knowledge base, to achieve the analysis of the results of the disease, and on this basis, to evaluate the effect of the relevant drugs for the treatment of mental diseases. The advantage of the construction of deep convolution neural network system in this study is that it effectively improves the induction, classification, and analysis efficiency of modern mental diseases using the algorithm, makes the disease screening means more comprehensive and informative, improves the screening accuracy, and reduces the consumption of doctors' human resources, which provides a theoretical basis for the future digitization of the medical industry.

The article "Construction and Drug Evaluation Based on Convolutional Neural Network System Optimized by Grey Correlation Analysis" was retracted in 2023. Reasons: unreliable results or conclusions; concerns about the data; concerns about the peer review; concerns about the citations.

## 2. Grey Correlation Analysis of Mental Illness Cases

### 2.1. Construction of Grey Correlation Analysis System

Grey relational analysis (GRA) is a commonly used analysis method, which is mostly used to count the influence of multiple factors on the results. The basic process is to determine the composition of reference data column and comparison data column, which reflects the degree of correlation between data. When using grey correlation analysis to solve the problems of comprehensive evaluation, it is necessary to calculate and analyze the subsequence and the parent sequence, which are changing with the events according to certain rules and on the basis of establishing the parent sequence, so as to get the degree of correlation between the two and draw a conclusion. The specific flow chart is shown in Figure 1 [29].

First of all, we need to be clear about the two basic sequences. The first is the sequence of specific behavior characteristics of the reaction process system, which is called reference sequence here. The other is the sequence that has a certain impact on the system behavior, which we call comparative sequence. The formula is as follows:

References sequence:

(1) $$\begin{array}{c} Y\left(k\right)|k=1,2,\ldots ,n. \end{array}$$

Comparison sequence:

(2) $$\begin{array}{c} X_{i}\left(k\right)|k=1,2,\ldots ,n,\;i=1,2,\ldots ,m. \end{array}$$

After defining these two sequences, we need to do some dimensionless processing on the data. The reason is that different dimensions in the system will have a certain degree of influence on the data in each factor column, which will interfere with our correct experimental results, so it is very necessary to carry out dimensionless data processing. We can do dimensionless processing by the following two methods.

First, initial value processing:

(3) $$\begin{array}{c} x_{i}\left(k\right)=\frac{x_{i}\left(k\right)}{x_{i}\left(1\right)},\;k=1,2,\ldots ,n;\;i=0,1,2,\ldots ,m. \end{array}$$

The second is the average processing:

(4) $$\begin{array}{c} x_{i}\left(k\right)=\frac{x_{i}\left(k\right)}{x_{i}},\;k=1,2,\ldots ,n;\;i=0,1,2,\ldots ,m. \end{array}$$

In the above two formulas (3) and (4), *k* represents the time, and *i* represents an eigenvalue in the comparison sequence.

The article "Construction and Drug Evaluation Based on Convolutional Neural Network System Optimized by Grey Correlation Analysis" was retracted in 2023. Reasons: unreliable results or conclusions; concerns about the data; concerns about the peer review; concerns about the citations.

After processing the data, we will calculate the correlation coefficient.

(5) $$\begin{array}{c} \zeta_{i}\left(k\right)=\frac{\underset{i}{\min}\underset{k}{\min}\left|y\left(k\right)-x_{i}\left(k\right)\right|+\rho \underset{i}{\max}\underset{k}{\max}\left|y\left(k\right)-x_{i}\left(k\right)\right|}{\left|y\left(k\right)-x_{i}\left(k\right)\right|+\rho \underset{i}{\max}\underset{k}{\max}\left|y\left(k\right)-x_{i}\left(k\right)\right|}. \end{array}$$

Note that

(6) $$\begin{array}{c} {△}_{i}\left(k\right)=\left|y\left(k\right)-x_{i}\left(k\right)\right|. \end{array}$$

Then

(7) $$\begin{array}{c} \zeta_{i}\left(k\right)=\frac{\underset{i}{\min}\underset{k}{\min}{△}_{i}\left(k\right)+\rho \underset{i}{\max}\underset{k}{\max}{△}_{i}\left(k\right)}{{△}_{i}\left(k\right)+\rho \underset{i}{\max}\underset{k}{\max}{△}_{i}\left(k\right)}. \end{array}$$

Among them,

(8) $$\begin{array}{c} \rho \epsilon \left(0,\infty \right). \end{array}$$

In these formulas, *ρ* is the resolution coefficient. When its value is smaller, the resolution of analysis will be larger. Generally, the value range is (0, 1). In general, we think that when *ρ* < 0.5463, the resolution of this case is the best, so it is usually *ρ*=0.5.

Next, we need to calculate the correlation coefficient. Because the correlation coefficient is the correlation degree value of the comparison sequence and the reference sequence at each time (that is, each point in the curve), it has more than one number, and the information is too scattered to facilitate the overall comparison. In order to make a better overall comparison, we need to integrate each point in the curve into a numerical value, that is, to calculate the average value, and reflect the correlation between the comparison sequence and the reference sequence on the basis of the average value [30]. The formula is as follows:

(9) $$\begin{array}{c} r_{i}=\frac{1}{n}\overset{n}{\underset{k=1}{\sum }}\zeta_{i}\left(k\right),\;k=1,2,\ldots ,n. \end{array}$$

Then, we compare the two values. If *r*_1_ < *r*_2_, the reference sequence *y* is more similar to the comparison sequence *x*_2_.

### 2.2. Analysis of Mental Illness Cases

The system includes medical document preprocessing module, which is used to clean up illegal characters in medical text big data, unify Chinese character encoding, and generate word table for word vector training. The word vector training module is used to read preprocessed medical texts. By training a deep convolutional neural network, the primary word vector is generated by optimizing the probability of the language model. The distributed semantic characteristics of medical information extraction module take the primary keyword as the starting point of the vector, using deep convolution neural networks, mapping the original data to hidden layer feature space, and finally, we use the full connection layer to map distributed features to a sample label space. Thus, the distributed semantic features in the medical field are generated for the risk assessment of mental diseases and the evaluation of drug efficacy.

The article "Construction and Drug Evaluation Based on Convolutional Neural Network System Optimized by Grey Correlation Analysis" was retracted in 2023. Reasons: unreliable results or conclusions; concerns about the data; concerns about the peer review; concerns about the citations.

We need to deal with the massive data of mental illness and build an evaluation system, which is widely applicable to the analysis of mental illness. The premise of this system is to process the existing data of mental illness according to the corresponding indicators. This study conducted a grey correlation analysis on the incidence rate of mental illness to explore the influencing factors of mental illness. Mental diseases are usually divided into schizophrenia, psychosexual disorders, and personality disorders. We analyzed the incidence rate of some mental disorders reported in a recent 5 years. We used the reported incidence rate as a reference sequence (*A*_0_) in the past years, taking schizophrenia, *A*_1_, *A*_2_, and *A*_3_ as the comparison sequence. We adopted the initial steps to carry out the dimensionless processing through the basic steps of grey correlation analysis and then calculated the correlation coefficients based on the normalized values after the treatment was processed [31]. The results are shown in Figure 2.

From Figure 2, we can analyze that the incidence rate of *A*_2_ mental illness in the past five years is relatively high in the three cases, which may be attributed to the changes in social and cultural development in recent years as the development of science and technology.

Next, we also analyzed the correlation between mental illness and patients' age, gender, height, weight, occupation, and income, as shown in the figure. It can be seen from Figure 3 that the incidence of mental illness has the highest correlation with the income of patients and the lowest correlation with gender.

There are many methods of factor analysis, such as regression analysis, including linear regression, multifactor regression, single factor regression, stepwise regression, nonstepwise regression, and so on. The above methods generally require a large amount of data, typical distribution, and large amount of calculation. Grey correlation analysis is based on the development trend of the process and the spatial distribution of related samples, in order to explain the correlation between the two. As shown in Figure 4, it is the error surface diagram after three repetitions of grey correlation analysis data calculation, and the error range is within the allowable value (*a* < 1).

The article "Construction and Drug Evaluation Based on Convolutional Neural Network System Optimized by Grey Correlation Analysis" was retracted in 2023. Reasons: unreliable results or conclusions; concerns about the data; concerns about the peer review; concerns about the citations.

The essence of factor analysis method is to analyze the geometry of the curve, judge whether the development trend is close or relevant from the correlation of geometry, and judge the specific value of correlation through the proximity of geometry, which can accurately reflect the dynamic development process between samples.

## 3. Construction of Convolution Neural Network System Optimized by Grey Correlation Analysis

In the field of deep learning, the first mock exam is the convolution neural network (CNN), which has been a major factor in the development of AI in recent years [32]. The advantage of this model is that it is necessary to extract features automatically and reduce the dimension of the feature based on convolution and pool operation.

As a special kind of neural network algorithm, the neurons in each layer of convolutional neural network have three dimensions, including width, height, and depth [33]. Convolution is based on a two-dimensional model, which has two numerical indicators of width and height, while depth refers to the dimension of active data volume in convolution network. The main flow of convolution neural network algorithm is shown in Figure 5. The data are transformed and analyzed through three dimensions and finally output to specific vector data through the output layer.

Convolutional neural network is mainly composed of input layer, convolution layer, relu layer, pooling layer, and fully connected layer. The deep learning algorithm for mental illness analysis and drug evaluation flow chart is shown in Figure 6.

Convolution layer is the core layer of convolution neural network, and most of the computation in the network is generated by convolution layer. Note the number of calculations not the number of parameters. The parameters of convolution layer are composed of a group of learning filters. The space for each filter is small (width and height), but the depth is the same as the input data. The formula for calculating the output size of any given convolution layer is as follows:

(10) $$\begin{array}{c} O=\frac{W-K+2P}{S}+1, \end{array}$$

where *k* is the filter size, *P* is the fill value, *S* is the step size, and *W* is the dimension of the input text matrix.

The actual output formula of the whole network is

(11) $$\begin{array}{c} O_{p}=F_{n}\left(F_{1}\left(XW_{1}\right)\right). \end{array}$$

The output of the current layer is expressed as

(12) $$\begin{array}{c} X^{1}=f^{1}\left(W^{1}WX^{1-1}+b^{1}\right). \end{array}$$

The activation function *F*_1_ is the correction linear unit, which is relu activation function

(13) $$\begin{array}{c} f^{1}=\max\left({\left(W^{1}\right)}^{T}X^{1},0\right). \end{array}$$

When dealing with some complex input problems, such as image processing, each neuron cannot perfectly link with the previous neuron. In this case, we need to transform the connection part of each neuron into a specific area in the part of the previous input data. This area is called the receiving domain, and the actual size of the receiving domain is a super parameter. In the depth direction, the size of the connection is always equal to the depth of the input.

The article "Construction and Drug Evaluation Based on Convolutional Neural Network System Optimized by Grey Correlation Analysis" was retracted in 2023. Reasons: unreliable results or conclusions; concerns about the data; concerns about the peer review; concerns about the citations.

In addition, the existence of receptive field also explains the specific structure of convolution layer in deep convolution neural network, in which each neuron has a certain connection with the input data sample, and how each neuron arranges with the corresponding input data needs to be clarified in this part. In general, there are three super parameters to control the output volume, including depth, step size, and zero fill. It can be calculated by inputting relevant data, including receptive field size (*F*), step size (*S*), number of filters (*K*), and number of zero padding (*P*) of neurons in convolution layer

(14) $$\begin{array}{c} W_{2}=\frac{W_{1}-F+2P}{S}+1,\\ H_{2}=\frac{H_{1}-F+2P}{S}+1. \end{array}$$

Generally speaking, when the step size *S* = 1, the value of zero padding is *P* = (*F* − 1)/2, which can ensure that the input and output data bodies have the same space size.

In the convolution layer, the number of parameters is generally regulated by the weight, and even in the same convolution layer, the weight of each receptive field may be different, which will lead to a huge amount of data in such a complex situation.

Usually, a pooling layer is periodically inserted between successive convolution layers. Its function is to gradually reduce the spatial size of the data body. In this way, the number of parameters in the network can be reduced, the cost of computing resources can be reduced, and the over fitting can be effectively controlled.

The corresponding formula in the convergence layer is as follows:

(15) $$\begin{array}{c} W_{2}=\frac{W_{1}-F}{S}+1,\\ H_{2}=\frac{H_{1}-F}{S}+1. \end{array}$$

There are two main differences between this method and the previous convolution size calculation. Firstly, there is no additional supplement in the pooling process; Secondly, the depth of pool remains unchanged.

The deep convolution neural network mainly uses the back propagation of the error function and uses the random gradient descent method to optimize and adjust the convolution parameters and deviations until the network converges or stops when the maximum number of iterations is reached. In this process of back propagation, it is usually necessary to compare different data samples with corresponding labels and then calculate the square error cost function to identify multiple categories of *c* categories and N training samples. The final output error function of the network is calculated by the following formula:

(16) $$\begin{array}{c} E^{N}=\frac{1}{2}\overset{N}{\underset{n=1}{\sum }}\overset{c}{\underset{k=1}{\sum }}{\left(t_{k}^{n}-y_{k}^{n}\right)}^{2}. \end{array}$$

BP algorithm is used to calculate the error function

(17) $$\begin{array}{c} \delta^{1}={\left(W^{l+1}\right)}^{T}\delta^{l+1}f^{\prime }\left(u^{\prime }\right), \end{array}$$

of which

(18) $$\begin{array}{c} u^{\prime }=W^{l}x^{l+1}+b^{l}. \end{array}$$

Using grey correlation analysis to optimize convolution neural network algorithm is an improved method, which can give full play to the advantages of convolution neural network algorithm. The improved main flow chart is shown in Figure 7.

The article "Construction and Drug Evaluation Based on Convolutional Neural Network System Optimized by Grey Correlation Analysis" was retracted in 2023. Reasons: unreliable results or conclusions; concerns about the data; concerns about the peer review; concerns about the citations.

## 4. Analysis of Experimental Results and Drug Evaluation

In the above experimental analysis, we set the structure and related parameters of the deep convolution network. The structure of deep convolution network is composed of two convolution layers and two subsampling layers, which are connected alternately; The number of characteristic graphs of the lower sampling layer is consistent with that of the corresponding convolution layer. We analyze and compare the accuracy rates of traditional CNN, preprocessed CNN, and improved CNN algorithm system based on GRA and test the error recognition rates of the three algorithms after iterating once, and the results are shown in Figure 8.

With the development of science and technology, many deep learning models are considered to be used in the research of medical industry and related drugs. Among them, deep convolution network with its unique advantages has gained a lot of attention, its unique advantage is that it is good at classifying massive and complex data streams into smaller and smaller information. This characteristic is the key reason why deep convolution neural network can produce the best results in dealing with many complex problems, including image classification and speech recognition. Then, the depth convolution neural network model can recognize nose, ears, and eyes by combining edges. Finally, the model can learn face recognition and other fields by combining these parts.

The prediction of drug-drug interaction (DDI) is a very challenging problem for pharmacology and clinical application. Drug-drug interaction refers to the connection and chemical interaction between two or more drugs under certain conditions, which may lead to unexpected side effects in the treatment process. In recent years, many reports also show the importance of the study of drug interactions. If we can predict DDI in advance, we can do this and provide the theoretical basis of neural network algorithm calculation for the drug treatment of mental diseases in the future.

The article "Construction and Drug Evaluation Based on Convolutional Neural Network System Optimized by Grey Correlation Analysis" was retracted in 2023. Reasons: unreliable results or conclusions; concerns about the data; concerns about the peer review; concerns about the citations.

There are several methods for DDI prediction. The first is molecular characterization, which mainly focuses on the feature learning of drug molecules. These methods are based on the same assumption that drug molecules with similar embedding representation will show similar DDI. If molecules A and B have similar molecular structures and so do their learning eigenvectors. If molecule A interacts with molecule C, it can be inferred that molecule B and molecule C have similar DDI. There are many methods to learn drug molecular features, such as one-dimensional smile sequence similar to text coding, such as traditional methods based on molecular descriptors or molecular fingerprint ECFP or methods based on 3D coordinate axis position information.

Another commonly used DDI prediction method is based on network embedding. By constructing various biological networks related to drugs, drugs are regarded as nodes in the network, and the relationship between potential edges, namely, DDI, is predicted by learning the embedded representation of nodes. There are many ways to establish the mapping relation network, such as matrix decomposition or constructing the objective relation into a matrix to solve. For example, random walk, choose a fixed path to walk in the graph to obtain more node features. The goal of these methods is to predict the label edge between drugs, but they only focus on a single DDI relationship and do not consider other links related to drugs.

The system preprocesses the electronic health documents of mental illness patients and builds a language model to transform the text into word vector. The distributed semantic features of clinical documents were extracted by deep convolutional neural network, and the long-term semantic correlation features were obtained by combining with deep grid long-term and short-term memory neural network, which could be used for the subsequent evaluation and analysis of the efficacy of related drugs in patients with mental illness.

In this study, we use the convolution neural network algorithm system optimized by grey correlation analysis to analyze the related drugs 1–4 for depression, which is an important treatment of mental illness. We can comprehensively judge the drug effect by comparing its six different clinical treatment indicators. The results are shown in Figure 9. It can be seen from the analysis of the results in Figure 9 that among the four drugs used for the treatment of depression, the scores generated by each clinical index are different, and the final comprehensive evaluation score can better reflect the effect of the drug in the clinical treatment process. From the results of this analysis, it can be seen that the comprehensive evaluation score of drug 1 is the best, followed by drug 3, followed by drug 4, and finally drug 2 has the lowest comprehensive evaluation score. Based on the above results, it can provide data theoretical guidance for the follow-up treatment of depression. This evaluation system provides more possibilities for improving the relevant medical means or drug combination.

The article "Construction and Drug Evaluation Based on Convolutional Neural Network System Optimized by Grey Correlation Analysis" was retracted in 2023. Reasons: unreliable results or conclusions; concerns about the data; concerns about the peer review; concerns about the citations.

## 5. Conclusion

In this study, a mental disease grey correlation analysis system and related drug evaluation system based on deep convolutional neural network were developed and constructed, which innovatively applied deep convolutional neural network to the analysis of mental diseases and the evaluation of related drugs, providing great convenience for the diagnosis and treatment of mental diseases. The establishment of this system can effectively improve the automation and intelligence of modern mental illness treatment process. In this article, the grey correlation analysis of the patient data was carried out, and then the construction of the optimized depth convolution neural network was done, combined with the medical knowledge base, to achieve the analysis of the results of the disease, and on this basis, to evaluate the effect of the relevant drugs for the treatment of mental diseases. The advantage of the construction of deep convolution neural network system in this study is that it effectively improves the induction, classification, and analysis efficiency of modern mental diseases by using the algorithm, makes the disease screening means more comprehensive and informative, improves the screening accuracy, and reduces the consumption of doctors' human resources, which provides a theoretical basis for the future digitization of the medical industry.

## Figures and Tables

**Figure 1:** Grey correlation analysis flow chart.

**Figure 2:** Correlation coefficient and correlation degree of each disease and reported incidence over the years.

**Figure 3:** The correlation between mental illness and influencing factors.

**Figure 4:** Grey correlation analysis data were used to calculate the error after three repetitions.

The article "Construction and Drug Evaluation Based on Convolutional Neural Network System Optimized by Grey Correlation Analysis" was retracted in 2023. Reasons: unreliable results or conclusions; concerns about the data; concerns about the peer review; concerns about the citations.

**Figure 5:** Convolutional neural network model diagram.

**Figure 6:** Deep learning algorithm for mental illness analysis and drug evaluation flow chart.

**Figure 7:** Algorithm flow chart of convolutional neural network system optimized by grey correlation analysis.

**Figure 8:** Error rate after iteration of the three algorithms: traditional CNN, preprocessed CNN, and improved CNN algorithm system based on GRA.

**Figure 9:** Comprehensive evaluation of drugs by clinical indicators.

## Data Availability

The data used to support the findings of this study are available from the corresponding author upon request.

## References

[1] Sarıgül M., Ozyildirim B. M., Avci M. (2019). Differential convolutional neural network. *Neural Networks*.

[2] Shan W., Li X., Yao H., Lin K. (2021). Convolutional neural network-based virtual screening. *Current Medicinal Chemistry*.

[3] Cai T., Zhao Z. (2020). Convolutional neural network-based surgical instrument detection. *Technology and Health Care*.

[4] Anwar S. M., Majid M., Qayyum A., Awais M., Alnowami M., Khan M. K. (2018). Medical image analysis using convolutional neural networks: a review. *Journal of Medical Systems*.

[5] Hochuli J., Helbling A., Skaist T., Ragoza M., Koes D. R. (2018). Visualizing convolutional neural network protein-ligand scoring. *Journal of Molecular Graphics and Modelling*.

[6] Matyushin D. D., Sholokhova A. Y., Buryak A. K. (2019). A deep convolutional neural network for the estimation of gas chromatographic retention indices. *Journal of Chromatography A*.

[7] Chantsalnyam T., Lim D. Y., Tayara H., Chong K. T. (2020). ncRDeep: non-coding RNA classification with convolutional neural network. *Computational Biology and Chemistry*.

[8] Xu S., Li R., Wang Y. (2020). Research and verification of convolutional neural network lightweight in BCI. *Computational and mathematical methods in medicine*.

[9] Bai Y.-t., Jin X.-b., Wang X.-y., Wang X.-k., Xu J.-p. (2020). Dynamic correlation analysis method of air pollutants in spatio-temporal analysis. *International Journal of Environmental Research and Public Health*.

[10] Bu F., He J., He J., Li H., Fu Q. (2020). Interval-valued intuitionistic fuzzy MADM method based on TOPSIS and grey correlation analysis. *Mathematical Biosciences and Engineering*.

[11] Li P., Ji Y., Wu Z., Qu S.-J. (2020). A new multi-attribute emergency decision-making algorithm based on intuitionistic fuzzy cross-entropy and comprehensive grey correlation analysis. *Entropy*.

[12] Bu F., He J., He J., Li H., Fu Q. (2020). Correction: interval-valued intuitionistic fuzzy MADM method based on TOPSIS and grey correlation analysis. *Mathematical Biosciences and Engineering*.

The article "Construction and Drug Evaluation Based on Convolutional Neural Network System Optimized by Grey Correlation Analysis" was retracted in 2023. Reasons: unreliable results or conclusions; concerns about the data; concerns about the peer review; concerns about the citations.

[13] Wang L., Yin K., Cao Y., Li X. (2018). A new grey relational analysis model based on the characteristic of inscribed core (IC-GRA) and its application on seven-pilot carbon trading markets of China. *International Journal of Environmental Research and Public Health*.

[14] Chowdhury S., Mainwaring P., Zhang L. (2020). Systematic review and meta-analysis of correlation of progression-free survival-2 and overall survival in solid tumors. *Frontiers in Oncology*.

[15] Bai L., Wang H., Shi C., Du Q., Li Y. (2017). Assessment of SIP buildings for sustainable development in rural China using AHP-grey correlation analysis. *International Journal of Environmental Research and Public Health*.

[16] Zhang J., Zhang A., Li J., Li F., Peng J. (2019). Gray correlation analysis and prediction on permanent deformation of subgrade filled with construction and demolition materials. *Materials*.

[17] Yasaka K., Akai H., Kunimatsu A., Kiryu S., Abe O. (2018). Deep learning with convolutional neural network in radiology. *Japanese Journal of Radiology*.

[18] Wang Z., Majewicz Fey A. (2018). Deep learning with convolutional neural network for objective skill evaluation in robot-assisted surgery. *International Journal of Computer Assisted Radiology and Surgery*.

[19] Su F., Shang H. Y., Wang J. Y. (2019). Low-rank deep convolutional neural network for multitask learning. *Computational Intelligence and Neuroscience*.

[20] Roy D., Panda P., Roy K. (2020). Tree-CNN: a hierarchical deep convolutional neural network for incremental learning. *Neural Networks*.

[21] Kaur R., Gholam Hosseini H., Sinha R. Deep convolutional neural network for melanoma detection using dermoscopy images.

[22] Kitrungrotsakul T., Han X.-H., Iwazzzto Y. (2019). VesselNet: a deep convolutional neural network with multi pathways for robust hepatic vessel segmentation. *Computerized Medical Imaging and Graphics*.

[23] Hu D., Peng F., Niu W. (2019). Deep convolutional neural network models for the diagnosis of thyroid cancer. *The Lancet Oncology*.

[24] Sumida I., Magome T., Kitamori H. (2019). Deep convolutional neural network for reduction of contrast-enhanced region on CT images. *Journal of Radiation Research*.

[25] Li Z., Zhou D., Wan L., Li J., Mou W. (2020). Heartbeat classification using deep residual convolutional neural network from 2-lead electrocardiogram. *Journal of Electrocardiology*.

[26] Lee S., Lee H., Myung W., Kim E. J., Kim H. (2018). Mental disease-related emergency admissions attributable to hot temperatures. *The Science of the Total Environment*.

[27] Tai A. M. Y., Albuquerque A., Carmona N. E. (2019). Machine learning and big data: implications for disease modeling and therapeutic discovery in psychiatry. *Artificial Intelligence in Medicine*.

The article "Construction and Drug Evaluation Based on Convolutional Neural Network System Optimized by Grey Correlation Analysis" was retracted in 2023. Reasons: unreliable results or conclusions; concerns about the data; concerns about the peer review; concerns about the citations.

[28] Isles A. R., Wilkinson L. S. (2008). Epigenetics: what is it and why is it important to mental disease?. *British Medical Bulletin*.

[29] Cui H., Guan Y., Chen H., Deng W. (2021). A novel advancing signal processing method based on coupled multi-stable stochastic resonance for fault detection. *Applied Sciences*.

[30] Deng W., Shang S., Cai X. (2021). Quantum differential evolution with cooperative coevolution framework and hybrid mutation strategy for large scale optimization. *Knowledge-Based Systems*.

[31] Li W., Zhang G., Yang X., Tao Z., Xu H. (2021). Sizing a hybrid renewable energy system by a coevolutionary multiobjective optimization algorithm. *Complexity*.

[32] Peng H., Han Y., Deng C., Wang J., Wu Z. (2021). Multi-strategy co-evolutionary differential evolution for mixed-variable optimization. *Knowledge-Based Systems*.

[33] Yao J., Chen Z., Liu Z. (2021). Improved ensemble of differential evolution variants. *PLoS One*.

